This article has been retracted.

# Malaria in urban, semi-urban and rural areas of southern of Gabon: comparison of the *Pfmdr 1* and *Pfcrt* genotypes from symptomatic children

**DOI:** 10.1186/s12936-016-1469-1

**Published:** 2016-08-18

**Authors:** Sydney Maghendji-Nzondo, Lady-Charlène Kouna, Gaël Mourembou, Larson Boundenga, Romeo-Karl Imboumy-Limoukou, Pierre-Blaise Matsiegui, Rella Manego-Zoleko, Bertrand Mbatchi, Didier Raoult, Fousseyni Toure-Ndouo, Jean Bernard Lekana-Douki

**Affiliations:** 1 Unité d’Evolution Epidémiologie Résistance Parasitaire (UNEEREP), Centre International de Recherches Médicales de Franceville (CIRMF), B.P. 769, Franceville, Gabon; 2 Département de Biologie, Université des Sciences et Techniques de Masuku, BP: 901, Franceville, Gabon; 3 Aix Marseille Université, URMITE, UM63, CNRS 7278, IRD 198, INSERM 1095, Marseille, France; 4 Département de Parasitologie-Mycologie Médecine Tropicale, Faculté de Médecine, Université des Sciences de la Santé, B.P. 4009, Libreville, Gabon; 5 Centre de recherches Médicales de la Ngounie, Fougamou, Gabon

**Keywords:** *Pfmdr1*, *Pfcrt*, Haplotype, ACT, Resistance, SNPs, Children, Gabon

## Abstract

**Background:**

Artesunate-amodiaquine (AS-AQ) and artemether-lumefantrine (AL) are first- and second-line treatments for uncomplicated *Plasmodium falciparum* malaria in Gabon. AL remains highly efficacious, but its widespread use has led to molecular selection of the NFD haplotype on *Pfmdr1* and K76 in *Pfcrt*. In this study, plasmodial infection characteristics and the distribution of the *Pfmdr1* and *Pfcrt* genotypes involved in reduced efficacy of artemisinin-based combination therapy (ACT) were investigated in four Gabonese localities.

**Methods:**

A cross-sectional study was conducted in the paediatric units of rural (Lastourville and Fougamou), semi-urban (Koula-Moutou) and urban (Franceville) areas. Malaria was diagnosed with the rapid diagnostic test Optimal-IT^®^ and confirmed by blood smear. *Pfmdr1* codons 86, 184 and 1246 and *Pfcrt* codon 76 were genotyped by PCR–RFLP and sequencing.

**Results:**

Among 1129 included children, the prevalence of plasmodial infection was 79.5 % at Lastourville, 53.6 % at Fougamou, 36.1 % at Koula-Moutou, and 21.2 % at Franceville. The prevalence was significantly higher among children over 60 months of age in both semi-urban (p = 0.01) and urban (p = 0.004) areas. The prevalence of *Pfmdr1* wild-type N86 differed significantly between Lastourville (57.8 %) and Koula-Moutou (45.4 %) (p = 0.039). No difference in 184F-carrying parasites was found between Lastourville (73.8 %), Fougamou (81.6 %), Koula-Moutou (83.2 %), and Franceville (80.6 %) (p = 0.240). The prevalence of wild-type D1246 was significantly different between Lastourville (94.1 %), Koula-Moutou (85.6 %) and Franceville (87.3 %) (p = 0.01). The frequency of wild-type K76 was not significantly different across the four sites: Lastourville (16.5 %), Fougamou (27.8 %), Koula-Moutou (17.4 %), and Franceville (29.4 %) (p = 0.09). The mixed genotypes were only found in Lastourville and Franceville. The NFD, YFD and NYD haplotypes were mainly Lastourville (46.6, 25.8, 14.0 %), Fougamou (45.5, 9.1, 42.4 %), Koula-Moutou (35, 6.7, 40.4 %), and Franceville (40.0, 16.0, 32.0 %).

**Conclusion:**

This study shows an increase in the prevalence of childhood plasmodial infection in Gabon according to the low socio-economic level, and a high frequency of markers associated with AL treatment failure. Close monitoring of ACT use is needed.

## Background

*Plasmodium falciparum* malaria is the most frequent parasitic infection worldwide, and is especially prevalent in sub-Saharan Africa. Anti-malarial drugs, such as chloroquine (CQ), amodiaquine (AQ) and sulfadoxine-pyrimethamine (SP) have lost some of their efficacy in malaria-endemic countries [1, 2]. The World Health Organization (WHO) has recommended the use of artemisinin-based combination therapy (ACT) to limit the drug resistance emergence since 2000. Cases of parasite resistance to artemisinin have now been detected in four countries of the Greater Mekong Sub-region: Cambodia, Myanmar, Thailand, and Viet Nam [3–5].

ACT treatment failures are linked to the selection of certain parasitic genotypic variants such as *Pfmdr1* N86 and *Pfcrt* K76 [6–8]. The *Pfmdr1* gene has been linked to resistance to CQ, AQ and mefloquine (MQ). Single nucleotide polymorphisms (SNPs) at codons 86 (N86Y), 184 (Y184F) and 1246 (D1246Y) confer reduced parasite sensitivity to various drugs, including ACT [6, 9–11]. For example, the *Pfmdr*-*1* Y86 mutation is associated with high-level CQ resistance when combined with the *Plasmodium falciparum* CQ resistance transporter (*Pfcrt*) T76 genotype [12, 13].

It has recently been shown that certain combinations of SNPs in the *Pfmdr*-1 gene, at codons 86, 184 and 1246, are emerging in areas where the ACT drug combination artemether-lumefantrine (AL) is widely used [14]. Certain *Pfmdr*-*1* haplotypes may be markers of emerging ACT tolerance [15]. Recent studies have shown that a combination of N86, 184F and D1246, creating the ‘NFD’ haplotype, reduces parasite susceptibility to AL, and that treatment with AL selects this haplotype [16, 17]. Other studies have shown that the combination of *Pfmdr*-*1* YYY haplotypes at codons 86/184/1246 are selected by AQ monotherapy and increase the risk of AQ failure [9, 10]. SNPs at positions 1034 and 1042 of *pfmdr1* have been shown to alter the drug-binding pocket in *Pfmdr1* [18] and are frequently found in Africa.

Gabon, in Equatorial Africa, is located in a hyperendemic area where malaria transmission is perennial. Resistance to CQ, AQ and sulfadoxine has already been described [19–21]. The 2003 consensus meeting in Gabon adopted ACT for the treatment of uncomplicated malaria and called for the withdrawal of CQ and other monotherapy. Artesunate-amodiaquine (AS-AQ) and AL were adopted as first- and second-line treatment for uncomplicated *P. falciparum* malaria, and quinine (QN) for severe malaria [22]. This led to a significant reduction in the paediatric malaria burden, in urban areas [23, 24]. ACT is currently implemented in urban and rural areas in Gabon, but few data on the prevalence of molecular markers of tolerance are available. Data from several rural areas are not available. Nothing is known of the use of preventative measures.

Franceville is a city with high levels of *P. falciparum* drug resistance, and in vitro reduced dihydroartemisinin (DHA) sensitivity has been reported [25]. It has recently been shown that the use of ACT selected the N86 genotype in Franceville [26]. This genotype is now suspected of being a marker of parasite tolerance of ACT [6, 11]. The purpose of the present study was to determine the general childhood malaria prevalence and to characterize the distribution of molecular genotypes of the *Pfmdr1* and *Pfcrt* genes involved in reduced *P. falciparum* clearance by ACT in four Gabonese localities.

## Methods

### Sites and study population

This study took place between May 2013 and July 2014 in four localities of southeast Gabon (Fig. 1): Fougamou, a rural area of Ngounie province; Lastourville and Koula-Moutou, rural and semi-urban areas of Ogooue-Lolo province; Franceville, the provincial capital of Haut-Ogooue. Blood samples were taken during outpatient paediatric consultations at the health centres of Fougamou and Lastourville, and the regional hospitals Paul Moukambi and Amissa Bongo in Koula-Moutou and Franceville, after obtaining informed consent from parents/guardians. The study population consisted of febrile children (≥37.5 °C or a history of fever less than 24 h before the consultation) aged from 6 to 168 months (15 years) in the outpatients’ departments of paediatrics. This age group was the most affected of the population by malaria. Children who did not fill the criteria and those among whom informed consent of parents or guardians was not obtained were excluded from the study. The study was approved by the Gabonese National Ethics Committee (no. 0023/2013/SG/CNE).

**Fig. 1:** Map of Gabon. Study sites are *underlined*

### Malaria diagnosis

The Optimal-IT^®^ rapid diagnostic test was used [27], and the sensibility and specificity test was 94 and 97 %. Preceding work in Gabon has shown that this test is a good tool for diagnosis of malaria [28]. Parasite load was determined on blood smears using the Lambarene method [29]. All blood smears were read by two independent technicians and quality control was done in 10 % of slides by a third reader. Fever and *P. falciparum* infection (1000 parasites per µl of blood) was considered to be malaria.

### Blood analysis

Routine haematological assays assessing the impact of malaria were done with an automated blood cell counter (STKS^®^, Coulter Corp, USA). Blood (5 ml) was collected in EDTA tubes. Plasma was stored at −20 °C and blood pellets were used for DNA extraction. Moderate anaemia was defined as a haemoglobin level between 5 and 10 g/dl, and severe anaemia as a haemoglobin level ≤5 g/dl.

### DNA extraction

DNA was extracted with the Omega Bio-Tek E.Z.N.A.1 method (Omega Bio-Tek, USA) according to the manufacturer’s protocol [26]. Briefly, 250 µl of blood, 25 µl of Omega Biotek (OB) protease (20 mg/ml), and 250 µl of lysis buffer were mixed and heated to 65 °C for 30 min before adding 260 µl of isopropanol. The mixture was transferred to a column and centrifuged at 10,000 rpm for 1 min. The column was washed twice at 13,000 rpm for 2 min, and DNA was eluted with 90 µL of sterile water preheated to 65 °C. DNA samples were kept at −20 °C until use.

### Amplification and genotyping of *Pfmdr1* at codons 86, 184 and 1246, and *Pfcrt* K76

Codons 86, 184, 1246, and 76 were amplified by nested PCR, using the primers listed in Extended Data [26, 30]. Five microlitre of DNA was amplified with 1X buffer, 0.8 µM each primer, 0.2 mM dNTP (Invitrogen^®^), 1.5 mM MgCl_2_ and 0.024 units of Taq DNA polymerase (Invitrogen^®^) using the following cycling programme: 5 min at 94 °C, then 35 cycles of 30 s at 94 °C, 45 s at 45 °C, 45 s at 72 °C, and a final extension step of 7 min at 72 °C. Codons 86, 184, 1246, and 76 of the *Pfmdr1* and *Pfcrt* genes were genotyped with a PCR–RFLP method as previously described [31]. The PCR products were digested with the restriction enzymes *Afl*III*, Dra*I*, Bgl*II and *Apo*I (New England Biolabs, UK) for SNPs N86Y, Y184F, D1246Y and K76T, respectively. To confirm the genotypes, double-strand sequencing of PCR products was performed with the Macrogen^®^ method. Sequences were analysed with MEGA6 software version 5.10 to identify specific SNP combinations. PCR products were detected by 2 % agarose gel electrophoresis.

### Statistical analysis

Epi-info version 3.3.2 (2005, CDC, Atlanta, USA) and STATA version 14.0 (Stata Corp, College Station, USA) were used for statistical analyses. Age was expressed as the mean and standard deviation (SD), and parasite density as the geometric mean (GMPD) and range. The Chi square test was used to compare categorical variables, and the non-parametric Kruskal–Wallis test, Pearson’s test or Fisher’s exact test for group comparisons, as appropriate. *P* values <0.05 were considered to indicate statistical significance.

## Results

### Study population

A total of 1129 children were included between May 2013 and July 2014. The general characteristics of the children are described in Table 1. The proportion of children aged between 6 and 60 months was significantly different from the proportion of children older than 60 months at all the sites (p < 0.001). Mean age was higher in the urban and semi-urban areas than in the rural area (p < 0.001). Haematological parameters [haemoglobin, white blood cells, red blood cells (Hb, WBC, RBC)] differed significantly between the rural (Lastourville) and urban areas (Franceville) (p < 0.01). Platelet counts differed significantly between the rural, semi-urban and urban areas (p < 0.001).

**Table 1:** Sociodemographic and biological characteristics of the included children by sites

	LTV	p	FGM	p	KMT	p	FCV	p				
	(N = 387)		(N = 98)		(N = 357)		(N = 280)					
General characteristics												
Sex ratio	1.2		1.2		0.9		1.1					
Mean temperature ± SD (°C)	38.4 ± 1.2		38.4 ± 1.1		37.8 ± 1.3		38.3 ± 1	0.0001				
Mean age ± SD (month)	47.3 ± 34.7		44.03 ± 39.1		53.7 ± 49.1		59.4 ± 37.5	0.0001				
Haemoglobin (g/dl)	9.4 ± 2.2		ND		9.7 ± 1.9		10 ± 1.7	0.0001				
WBC (×10^3^/µl)^a^	10.3 ± 6.3		ND		9.4 ± 3.9		8.9 ± 6.2	0.0009				
RBC (×10^6^/µl)^b^	3.5 ± 0.9		ND		4.0 ± 0.8		4.5 ± 2.7	0.0001				
Platelet (×10^3^/µl)	144.1 ± 121.6		ND		239.6 ± 134.9		255.3 ± 131.2	0.0001				

Age group	Prevalence of malaria infection [%; (n/N)]											
<60 months	77.6 (211/272)		50.7 (36/71)		31.6 (72/228)		15.1 (23/152)					
>60 months	84.2 (80/95)		58.3 (24/24)		46.1 (53/115)		28.7 (31/108)					
p	0.2		0.68		*0.01*		*0.004*					

Prevention measures	Number of children (%, n)											
	Uninfected	Infected	p	Uninfected	Infected	p	Uninfected	Infected	p	Uninfected	Infected	p
Bed net	66.7 (48)	42.7 (126)	*0.004*	71.1 (32)	79.2 (42)	0.48	66.2 (147)	64.6 (82)	0.84	53.3 (113)	48.2 (27)	0.59
Insecticides	13.9 (10)	14.1 (40)	0.88	21.9 (9)	18.9 (10)	0.91	30.2 (67)	27.8 (35)	0.72	39.3 (83)	33.9 (19)	0.55
Received an IEK on malaria	28.6 (20)	23.7 (67)	*0.02*	95.2 (40)	92.2 (47)	0.85	73.2 (161)	74.0 (91)	0.97	65.4 (138)	61.8 (34)	0.73

*IEK* information, education and knowledge; *LTV* Lastourville; *KMT* Koula-Moutou, *FGM* Fougamou, *FCV* Franceville; *ND* undetermined

^a^White blood cell

^b^Red blood cell

### *Plasmodium* characterization

The prevalence of *Plasmodium* infection was, respectively, 79.5, 53.6, 36.1, and 21.2 % at Lastourville, Fougamou, Koula-Moutou, and Franceville. The overall prevalence was higher in rural areas (74.2 %; n = 351/473) than in semi-urban and urban areas (p < 0.001).

As shown in Table 2, *Plasmodium*-infected children were older than uninfected children at Lastourville, Koula-Moutou and Franceville. The Kruskal–Wallis test showed a significant difference (p < 0.001) in mean age between the rural, semi-urban and urban areas.

**Table 2:** Biological characteristics of uninfected versus infected children by site

Characteristics	LTV			FGM			KMT			FCV		
	Uninfected	Infected	p	Uninfected	Infected	p	Uninfected	Infected	p	Uninfected	Infected	p
Malaria prevalence (%)		77.3			53. 6			36.1			21.2	
Sex ratio	1.3	1.1	0.543	1.3	1.1	0.709	0.9	0.8	0.325	1.2	0.7	0.101
Mean temperature ± SD (°C)	38.1 ± 1.2	38.5 ± 1.2	*0.011*	37.7 ± 0.9	38.6 ± 1.3	*0.0007*	37.6 ± 1.2	38.0 ± 1.0	*0.003*	38.3 ± 0.9	38.5 ± 1.0	0.38
Mean age ± SD (monthS)	45.8 ± 35.6	50.0 ± 35.0	*0.002*	40.0 ± 43.3	44.0 ± 39.0	0.22	49.7 ± 38.2	60.8 ± 43.5	*0.019*	54.1 ± 37.1	78.7 ± 34.0	*2.04 × 10* ^−*5*^
Haemoglobin (g/dl)	9.6 ± 2.3	9.4 ± 2.2	0.506	ND	ND		10.1 ± 1.7	8.9 ± 2.0	<*0.001*	10.3 ± 1.5	9.8 ± 2.0	0.151
WBC (10^3^/µl)	14.8 ± 11.4	9.5 ± 5.5	*0.005*	ND	ND		9.9 ± 4.3	8.5 ± 3.1	*0.003*	9.4 ± 6.7	6.9 ± 3.6	*0.001*
RBC (10^6^/µl)	3.7 ± 1.2	3.4 ± 0.9	0.103	ND	ND		4.2 ± 0.8	3.7 ± 0.7	<*0.001*	4.6 ± 2.9	4.1 ± 0.8	*0.020*
Platelets (10^3^/µl)	290.3 ± 157.7	115.3 ± 90.5	<*0.001*	ND	ND		296.4 ± 128.3	146.1 ± 85.7	<*0.001*	266.9 ± 117.3	179.9 ± 143.3	*0.001*
Parasitaemia (p/µl)^a^		7510 (56–571,200)			34,020 (172–490,200)		4535 (36–38,880)				8574 (420–453,600)	*0.0001*

*LTV* Lastourville; *FGM* Fougamou; *KMT* Koula-Moutou; *FCV* Franceville; *ND* undetermined

^a^Geometric mean parasitaemia (min–max)

Haemoglobin, red blood cell, white blood cell, and platelet values were lower in *Plasmodium*-infected children than in uninfected children (p < 0.001) in the semi-urban area (Koula-Moutou). The Kruskal–Wallis test showed a significant difference in mean haematological values (Hb, WBC, RBC, platelets) between rural, semi-urban and urban areas (p < 0.001).

Finally, a significant difference in mean parasitaemia was observed between Lastourville and Koula-Moutou (p < 0.001), between Lastourville and Fougamou (p = 0.011), Koula-Moutou and Fougamou (p < 0.001), between Koula-Moutou and Franceville (p = 0.006), and between Franceville and Fougamou (p = 0.006). The prevalence of plasmodial infection is summarized in Table 1 according to the age group (<60 and >60 months).

### Preventive measures

Univariate and multivariate analysis showed no association between the use of preventive measures and malaria prevalence, excepted at Lastourville, where the use of bed nets was associated with a lower prevalence [p < 0.001; OR 0.37 (0.22–0.64)] (Table 1).

### Seasonality

In Gabon the year begins with a short dry season between January and February, then a long rainy season between March and May, followed by a long dry season between June and September, and finally a short rainy season between October and December. Figure 2 shows variations of malaria transmission during the period of study. Data showed that the frequency of plasmodial infection was significantly different across the seasons at all sites (p < 0.001).

**Fig. 2:** Temporal distribution of plasmodial infection. Short rainy season (*short blue line*), long rainy season (*large blue line*), short dry season (*short yellow line*), and long dry season (*large yellow line*)

### Prevalence of SNPs at codons 86, 184, 1246 of *pfmdr1* and *codon* 76 of *Pfcrt*

The distribution of SNPs at codons 86, 184, 1246 of *Pfmdr1* and codon 76 of *Pfcrt* is summarized in Table 3 for each locality.

**Table 3:** Molecular markers and haplotype prevalence

Prevalence by sites [%; (n/N)]							
Genes	Codons	Genotypes	LTV	FGM	KMT	FCV	p
*Pfcrt*							
SNPs	76	K	16.5 (33/200)	27.8 (10/36)	17.4 (20/115)	29.4 (15/51)	0.09
		K/T	10.5 (21/200)	0.0 (0/36)	0.0 (0/115)	17.6 (9/51)	ND
	86	N	57.8 (144/249)	51.2 (21/41)	45.4 (49/108)	62.2 (23/37)	0.12
		N/Y	10.4 (26/249)	17.1 (7/41)	17.6 (19/108)	5.4 (2/37)	0.10
	184	Y/F	0.0	0.0	0.0	0.0	ND
		F	73.8 (175/237)	81.6 (31/38)	83.2 (84/101)	80.6 (25/31)	0.24
	1246	D	94.1 (255/271)	100.0 (32/32)	85.6 (95/111)	87.3 (48/55)	ND
		D/Y	3.3 (9/271)	0.0 (0/32)	12.6 (14/111)	9.1 (5/55)	ND
*pfmdr1*							
Haplotypes	86/184/1246	NFD	46.6 (110/236)	45.5 (15/33)	35.0 (31/89)	40.0 (10/25)	0.28
		NYD	14.0 (33/236)	9.1 (3/33)	6.7 (6/89)	16.0 (4/25)	ND
		YFD	25.8 (61/236)	42.4 (14/33)	40.4 (36/89)	32.0 (8/25)	*0.03*
		YYD	8.5 (20/236)	3.0 (1/33)	4.5 (4/89)	4.0 (1/25)	ND
		NFY	1.3 (3/236)	0.0	6.7 (6/89)	0.0	ND
		NYY	0.0	0.0	4.5 (4/89)	4.0 (1/25)	ND
		YYY	1.7 (4/236)	0.0	2.2 (2/89)	0.0	ND
		YFY	2.1 (5/236)	0.0	0.0	4.0 (1/25)	ND

*ND* p undetermined; *LTV* Lastourville; *FGM* Fougamou; *KMT* Koula-Moutou; *FCV* Franceville

The prevalence of wild-type N86 *Pfmdr1* was significantly different between Lastourville and Koula-Moutou (p = 0.03). The frequency of wild-type and mixed genotypes combined (N86 + 86 N/Y) was similar at all four sites (p = 0.22). No difference in the proportion of 184F-carrying parasites was found (p = 0.24). The prevalence of wild-type D1246 was significantly different between Lastourville and Koula-Moutou (p = 0.01). The frequency of wild-type and mixed genotypes combined (D1246 + 1246D/Y) was: Lastourville (97.4 %), Koula-Moutou (98.2 %), Franceville (96.4 %). Mixed-genotype D1246/Y1246 infections were infrequent with a significant difference between Lastourville and Koula-Moutou (p = 0.001).

Concerning the *Pfcrt* gene, the frequency of wild-type K76 was not significantly different across the four sites (p = 0.09). The frequency of mixed genotypes 76KT was not significantly different between Lastourville and Franceville (p = 0.244). The proportion of the mutated genotype (T76) was significantly different across the four sites (p = 0.001). The difference was more marked between Lastourville (73.0 %) and Fougamou (72.2 %) (p = 0.009) and between Fougamou and Koula-Moutou (82.6 %) (p = 0.001). The difference was no longer significant (p = 0.100) when the mixed genotype (KT) was included [Lastourville (83.5 %), Fougamou (72.2 %), Koula-Moutou (82.6 %), Franceville (70.6 %)]. The proportions of mixed genotypes did not differ between Lastourville and Franceville (p = 0.467).

### Haplotype distribution

The haplotypes were compared on a three-codon basis at each site, and mixed-genotype infections were included in the analysis (Table 3). Haplotypes NFD, NYD and YFD were most prevalent at Lastourville and haplotypes NFD and NYD were most prevalent at Fougamou, Koula-Moutou and Franceville. The prevalence of haplotype YFD was significantly different across the four sites: (p = 0.03). This difference was most marked between Lastourville and Koula-Moutou (p = 0.02). Minor haplotypes included YYD, NYY, YYY, NFY, and YFY.

## Discussion

This study shows that the prevalence of malaria in Gabon differs significantly according to local economic status, confirming previous data [32]. Malaria prevalence has remained stable in Franceville since 2011 [24]. This study confirmed that transmission is perennial in Gabon. In rural areas, anti-malarial drugs are under-used despite the availability of ACT. Poor socio-economic conditions and inadequate knowledge of malaria could contribute to the high prevalence of malaria in rural areas. Indeed, the study revealed that bed net use and knowledge of malaria were associated with a lower prevalence in Lastourville. These results are consistent with previous data from Franceville, where bed nets were found to contribute to malaria prevention (JBL-D, pers. comm.).

Data revealed no link between preventive measures and malaria prevalence in Fougamou, Koula-Moutou or Franceville, possibly because bed net use was very high overall. Environmental conditions could also contribute to maintaining a high level of malaria transmission observed in the study sites, as previously reported in Nigeria [33]. Lastourville, Fougamou, Koula-Moutou, and Franceville are crossed by rivers that favour *Anopheles* breeding and proliferation. Children over 5 years old were most likely to contract malaria in urban areas, in keeping with results from Oyem (a semi-urban area in northern Gabon), Melen (a suburb of Libreville) and Port-Gentil [34]. Surprisingly, no effect of malaria on the haemoglobin level was found, except at Koula-Moutou. In contrast, malaria was associated with significantly lower WBC and platelet counts.

It was found that ACT implementation has led to an increase in the prevalence of *P. falciparum* genotypes N86, 184F and D1246 in both rural and urban areas of Gabon. This is consistent with previous data from Gabon showing a significant increase in the prevalence of wild-type N86 at Oyem and Franceville [6, 9–11, 25, 26, 35]. Other studies in several African regions have shown similar genotype selection [7, 10–12]. Datas indicate a risk of diminished *P. falciparum* sensitivity to AL, as reported in Tanzania where the wild-type N86 and 184F *Pfmdr1* genotypes were associated with an increased risk of AL treatment failure [10, 13]. These genotypes were also selected on re-infection after AL treatment [11]. The high prevalence of SNPs associated with decreased sensitivity to ACT observed here suggests that these latter drugs are widely used in Gabon. One reason of increased prevalence of N86 and D1246 may be that SNPs associated with AQ resistance (Y86 and Y1246) have a higher fitness for parasites than N86 and D1246 [36], which would affect the selection pattern under different drug pressure. Another reason for change in prevalence of genotypes associated with CQ resistance could be the complete withdrawal of this drug as reported in Malawi [37]. Data founded show that NFD and YFD were the most prevalent haplotypes at each of the four study sites. NYD and YYD were the least prevalent and NFY, NYY, YYY, and YFY were not found at any of the sites (Table 3).

The findings are in keeping with those of a study from Maputo, where significant selection of NFD and NYD was observed 5–7 years after implementation of ACT in Mozambique [38]. In a study conducted in Tanzania, haplotype analysis showed a trend towards decreased lumefantrine susceptibility, in the order of NFD, NYD, YYY, and YYD [8]. This suggests gradual acquisition of tolerance, starting with N86, followed by the combination of N86 + D1246 and, thereafter, the combination of N86 + 184F + D1246 [8]. In Nigeria, the *Pfmdr1* haplotype of NFD was selected in recrudescence samples after AL treatment, suggesting that this haplotype conferred a fitness advantage in case of AL pressure [17]. Other studies of African samples support the selection of the NFD haplotype by AL [11, 39], while YYY is selected by AQ or CQ [10, 11, 40–42]. The study confirms the effective withdrawal of monotherapy. It has been shown that parasites carrying the *pfmdr1* NFD haplotype after AL treatment are able to re-infect patients with lumefantrine blood concentrations 15-fold higher than for parasites carrying the YYY haplotype [8]. This could explain the selection of NFD in Gabon. The high prevalence of NYD found here is consistent with reports of the selection of this haplotype in other regions after the introduction of AL [38, 43]. Data from Zanzibar showed that NYD was selected after AS-AQ implementation [36].

Selection of *Pfcrt* K76 was reported after the implementation of ACT [44]. In the present work, the prevalence of wild-type K76 was higher than previously reported in Lambarene and Franceville, showing the increase in this genotype after long-term use of ACT [26, 45]. This confirms that the increase in the prevalence of K76 after implementation of ACT occurs more slowly than the increase in N86 [6, 11]. Despite the significant increase in K76, its prevalence remains low. This could be explained by the late implementation of ACT in rural areas, even though ACT was already available in Gabon.

Mutations associated with artemisinin resistance in the K13 propeller gene (PF3D7_1343700 or PF13_0238) were not investigate in the study. Previous studies of samples from Gabon and other sub-Saharan African countries did not show the presence of mutations (C580Y, R539T, Y493H) incriminated in in vivo artemisinin resistance in Southeast Asia [46].

## Conclusion

This study shows an increase of the prevalence of plasmodial infection in Gabonese children, according to low socio-economic level. An age inversion of the population at risk in urban areas was found. A increase in the frequency of *Pfmdr1* haplotypes NFD, YFD and NYD in both rural and urban areas was observed. Also, a gradual increase in the frequency of the *Pfcrt* wild-type allele K76 in Franceville, 10 years after introduction of ACT in Gabon. Consequently, there is an urgent need to re-inforce strategies against malaria in both urban and rural settings, and to monitor ACT.

## Abbreviations

*Pfmdr1*: *Plasmodium falciparum* multidrug resistance 1
*Pfcrt*: *Plasmodium falciparum* chloroquine resistance transporter
AS-AQ: artesunate-amodiaquine
AL: artemether-lumefantrine
CQ: chloroquine
AQ: amodiaquine
ACT: artemisinin-based combination therapy
GMPD: parasite densities as geometric means
DNA: deoxyribonucleic acid
dNTP: nucleoside triphosphate
IEK: information, education and knowledge
CHRAB: Amissa Bongo Regional Hospital Centre
SP: sulfadoxine-pyrimethamine
MQ: mefloquine
SD: standard deviation
SNP: single-nucleotide polymorphism
DHA: dihydroartemisinin
